# Managing Anxiety Related to Anaphylaxis in Childhood: A Systematic Review

**DOI:** 10.1155/2012/316296

**Published:** 2011-10-05

**Authors:** Katharina Manassis

**Affiliations:** Department of Psychiatry, The Hospital for Sick Children, University of Toronto, 555 University Avenue, Toronto, ON, Canada M5G 1X8

## Abstract

*Objectives*. This paper reviews the relationship between anxiety and anaphylaxis in children and youth, and principles for managing anxiety in the anaphylactic child and his or her parents. *Methods*. A review of the medical literature (Medline) was done using the keywords “anxiety,” “anaphylaxis,” and “allergy,” limited to children and adolescents. Findings were organized into categories used in the treatment of childhood anxiety disorders, then applied to managing anxiety in the anaphylactic child. *Results*. Twenty-four relevant papers were identified. These varied widely in methodology. Findings emphasized included the need to distinguish anxiety-related and organic symptoms, ameliorate the anxiety-related impact of anaphylaxis on quality of life, and address parental anxiety about the child. *Conclusion*. Children with anaphylaxis can function well despite anxiety, but the physical, cognitive, and behavioral aspects of anxiety associated with anaphylactic risk must be addressed, and parents must be involved in care in constructive ways.

## 1. Introduction

Anxiety symptoms are common in children with anaphylactic conditions and in their parents. Children with anxiety disorders are at increased risk for allergies, including those associated with anaphylaxis [1], and anaphylaxis itself can provoke anxiety. Given the life-threatening nature of anaphylaxis, this anxiety is understandable especially within the first few months after diagnosis or after a reaction. Some anxiety in the face of anaphylaxis may even be adaptive, as anxious children are less likely to take risks with respect to their anaphylactic conditions than children who are not anxious [2]. 

In some cases, however, anxiety becomes debilitating and imposes unnecessary restrictions on the anaphylactic child's life, preventing the child from engaging in important daily activities at home, at school, or socially. Anxiety associated with such daily impairment is not considered normative [3]. For example, a child with an insect sting allergy might completely avoid the outdoors; a child with a severe food allergy might follow an overly restrictive diet or avoid friends' homes for fear of encountering an allergen; a young anaphylactic child might refuse to stay at school without a parent for fear of having a reaction there. Prominent symptoms of anxiety (e.g., hyperventilation or blushing) may also mimic anaphylactic reactions, often resulting in further anxiety and impairment [4–6]. 

Anxiety that is persistent, extreme, and results in restriction of activities that is not medically warranted must be addressed in order to return the child to a normative developmental course. Few guidelines exist on how to do this. Therefore, this paper reviews studies focusing on the relationship between anxiety and anaphylaxis in children and key clinical recommendations related to managing anxiety in the child and his or her parents. 

## 2. Materials and Methods

A review of the medical literature (Medline Search) was done using the keywords “anxiety” and “anaphylaxis,” limited to papers focusing on children and adolescents. The search yielded 17 papers, but 6 were excluded: 4 did not investigate any aspect of children's or parents' anxiety; 2 were reviews that did not contain new data. The remaining 11 papers were deemed relevant to this paper. These varied widely in methodology, but none were excluded for methodological reasons, given the paucity of studies. Scrutiny of these papers revealed additional citations that used the term “severe allergy” rather than anaphylaxis. Therefore, the original search was repeated using the term “allergy” instead of anaphylaxis, but only those papers that included children who might have anaphylactic reactions (mainly food and insect sting allergies) were included. This strategy yielded 13 additional papers, resulting in a total of 24 papers. Key findings and recommendations from each of these papers are summarized in Table 1. 

For the discussion, findings and recommendations were then further organized in relation to physiological, cognitive, behavioral, or parental aspects of anxiety. This was done because psychological interventions developed for children with anxiety disorders (e.g., cognitive behavioral therapy [7]) generally target these aspects. Focusing on these aspects allowed concepts relevant to interventions developed for childhood anxiety disorders to be applied to the special challenge of ameliorating anxiety in the context of pediatric anaphylaxis. 

## 3. Results and Discussion

Findings and interventions relevant to four aspects of anxiety (physiological, cognitive, behavioral, and parental), derived from the literature on pediatric anaphylaxis and on treatment of childhood anxiety disorders, will now be described. Successful management of anxiety in the anaphylactic child usually requires emphasis on those aspect(s) which predominate in a given child or family. 

### 3.1. Physiological Aspects of Anxiety

Recurrent, unexplained flushing [4], asthmatic attacks [6], anxiety-related syncope, and anxiety attacks [5] can all be mistaken for anaphylactic reactions in children and youth. For example, hyperventilation associated with anxiety can often cause tingling in the lips and extremities, prompting food allergic children to fear that they have come in contact with an allergen. Anxiety reactions that mimic anaphylaxis have also been noted during large-scale vaccination campaigns [5]. Education of children, families, school personnel, and public health providers is therefore important to improve their ability to distinguish anxiety symptoms from those of anaphylaxis, ensuring appropriate treatment [4–6]. When there is doubt, it is prudent to err on the side of caution and treat for anaphylaxis. However, when there are recurrent reactions in situations where the risk of allergen exposure is low, an anxious etiology should be suspected.

Children who become anxious in response to having an anaphylactic condition can often benefit from learning relaxation techniques such as slow, deep breathing, or progressive muscle relaxation (reviewed in [8]). These techniques must be practiced daily for a few weeks at nonanxious times (e.g., at bedtime) in order to become usable at anxious times. “Box breathing” is a particularly useful technique for reducing hyperventilation. In this technique, the child breathes in four stages and draws the sides of a box with his or her index finger in the process. These stages include breathing in, holding the breath, breathing out, and waiting for the next breath. The child is asked to count to 3 at each stage before moving on to the next, then count to 4 at each stage, and so on until breathing slowly. 

When anxiety symptoms subside, it is important to return the child quickly to his or her usual daily activities [8]. This practice has two benefits: it distracts the child from focusing further on any remaining symptoms, and it prevents reinforcement of avoidant behaviors that exacerbate anxiety in the long run. For example, if the child experiences anxiety symptoms at school, he or she can be helped to calm down by an adult in the school office, and then returned to class after a few minutes. Calling parents to come and remove the child from school is generally not helpful and may promote school avoidance. Of course, if there is a possibility of a true anaphylactic reaction, emergency medical services should be contacted.

### 3.2. Cognitive Aspects of Anxiety

Nut allergic children report a lower quality of life than their peers, and even than diabetic children [9, 10]. Children with anaphylactic conditions are especially vulnerable to worry and psychological distress relative to those with less severe allergies [11–13]. Separation anxiety is a particular concern in this population [14]. 

As mentioned above, some worry about having an anaphylactic reaction is natural and may be protective [2]. Unlike ordinary worries of childhood about low-risk events (e.g., worries about tests or examinations), worries about anaphylaxis focus on a life-threatening, high-risk event. Reassurance focused on minimizing this risk is therefore not helpful. Instead, reassurance must focus on the child's own ability to manage the risk. Education of the child and his or her parents about the degree of risk in various situations with emphasis on what the child can do to increase safety is an important first step towards reducing anxiety [2, 5, 14–22]. Then, the child should be engaged as a participant in a clear, concise plan for managing anaphylactic risk [22]. Such participation generally reduces children's sense of helplessness when living with an anaphylactic condition [14]. 

Young children may be limited in their ability to manage anaphylactic risk, as they are highly dependent on adults. However, they can still be engaged in practices that improve environmental safety (e.g., reminding people to read product labels; eliminating allergens from the home environment) [14]. Knowing when to ask an adult for help is another important skill for the young allergic child. Consistency in allergy management between environments (e.g., ensuring that the school and extended family members take the same precautions that the parents take) may further reduce the child's anxiety, as anxious children are typically reassured by predictability [7]. 

Adolescents, on the other hand, are often vulnerable to peer pressure and may cognitively minimize their allergic risk [15, 19]. High-risk behaviors with respect to anaphylaxis are particularly common among adolescents expressing little concern about their condition and among adolescents in social situations involving peers [19]. Inability to remember an anaphylactic reaction may also contribute to risk taking in adolescents [15]. Allergic youth with high health competence with respect to their condition, however, reported greater anxiety than those with low health competence [17] suggesting that education about anaphylaxis may result in a more realistic assessment of risk. Akeson and colleagues [15] have also emphasized the need to regularly review precautions and emergency management with adolescents in order to facilitate the transition from parental to self-management of anaphylactic risk.

Some aspects of the medical management of anaphylaxis can also affect children's and parents' anxiety. For example, use of epinephrine injectors has been found to reduce food allergic children's anxiety [9, 10]. On the other hand, children allergic to yellow jacket stings were found to be less anxious after venom immunotherapy than before, but continued to be anxious if given an epinephrine injector without immunotherapy [23]. Parental anxiety has been found to decrease after food challenges, regardless of challenge results [24].

### 3.3. Behavioral Aspects of Anxiety

Behavioral aspects of anxiety usually consist of unnecessary avoidance of certain situations or excessive clinginess with parents [14, 21, 25]. For example, some children with food allergies severely restrict food intake beyond what is medically necessary, adversely affecting their weight and nutrition [21], and some children anaphylactic to insect stings avoid all outdoor activities [13]. Other children continue to avoid certain foods despite a negative food challenge to those foods [25]. Repeating food challenges is reassuring in some but not all cases [25].

To begin to address unnecessary avoidance, obtain a detailed account of regularly avoided situations or foods (e.g., a 24-hour food recall) [21] or of situations where the child relies excessively upon his or her parents. Then, encourage daily practice approaching these situations or foods in small steps, beginning with a step that the child considers relatively easy (reviewed in [26]). In the case of food restriction, for example, the child may be involved in food preparation to increase confidence before being asked to eat a food that makes him or her anxious [21]. If a child with insect sting anaphylaxis avoids the outdoors, going outdoors in the winter (i.e., when there are no flying insects about) may be an easy first step. Although such practice is initially anxiety provoking, it results in cognitive desensitization to the feared stimulus, reducing anxiety over time [7]. If the child insists on parental accompaniment in this process, it is usually wise to allow it initially but then fade parental support gradually as the child gains confidence. Practice sessions should be long enough for the child's anxiety to peak and then begin subsiding (usually at least 20 minutes), as premature escape from the situation interferes with desensitization. 

To motivate the child's participation, it is often helpful to chart progress, providing praise and points or stickers for every attempt (reviewed in [26]). Providing a small reward every five or every ten points can increase motivation further. Adolescents may respond better to an extra privilege (e.g., extra “screen time” for their favorite computer activities; a little extra time to stay out with friends) than a tangible reward. Nutritional and/or behavioral guidelines may be needed for parents in order to optimize their participation in the child's anxiety desensitization program [21]. 

After a child becomes confident with the first step, he or she can begin practicing a step that is just slightly more anxiety provoking, with additional incentives for doing so if needed. Having mastered that step, the child then continues with further steps until there are no longer any situations or foods that are being unnecessarily avoided [7, 26]. 

### 3.4. Parental Aspects of Anxiety

Most authors cited in Table 1 noted anxiety in the parents of children with anaphylactic conditions, though some suggest that study recruitment may be somewhat biased towards more anxious parents [27]. Nevertheless, parental anxiety is common enough in this population that at least two relevant questionnaires have recently been developed and evaluated for parents of allergic children [12, 28]. Lebovidge and colleagues [12] developed a screening tool to identify parents of allergic children who are most vulnerable to anxiety. DunnGalvin and colleagues [28] suggest using The Food Allergy QoL-Parent Form to assess health-related quality of life in parents of food allergic children, including parental anxiety. Parents of food allergic children report that their child's allergy has a substantial impact on their quality of life [18, 20]. In one study this impact was reported as greater than that of having a child with rheumatological disease [18]. 

Studies of parental anxiety concluded that those whose children had multiple allergies or had anaphylaxis were most anxious [2, 12]. Consistent with these findings, adolescents with anaphylaxis reported more parental overprotection than those with less severe allergies [11]. Mothers may be especially vulnerable to anxiety about the child, as much of the management of children's allergies typically falls to their mothers [14]. Professionals, however, may also suffer excessive anxiety in response to even a remote risk of anaphylaxis. For example, family practitioners in Ireland frequently hospitalize children with egg allergies for routine vaccinations, even though this is not considered medically necessary [29]. 

Recommendations for addressing excessive parental anxiety include ongoing education and advice about realistic versus unrealistic risks (endorsed by all authors in this paper), especially in the form of clear, concise materials for families [22]; acknowledgment of psychological distress in families [11]; tailored information for families of adolescents to inform the transition from parental to self-management of allergy [14, 15]; recognizing patterns of family adaptation after an anaphylactic event [2], including the fact that anxiety in the first few months is normative; providing guidance for parents regarding optimal use of consumer organizations [16]; providing epinephrine injectors and instruction on how to use them to families of food allergic children with anaphylactic risk [9, 10]; providing venom immunotherapy to children with insect sting anaphylaxis [13, 23]; offering more peanut-free products for children with peanut allergy [18]; advocating for food labeling and public awareness of severe allergies and anaphylaxis [20, 22]. 

Working with anxious parents of children with anaphylactic conditions can be frustrating for professionals, especially when parents are difficult to reassure. However, it is important to enlist parents as allies in managing the child's allergy and to emphasize their ability to ensure safety, to model healthy coping, and to promote healthy coping in their child (reviewed in [8]). Putting oneself in the parents' shoes is often helpful, as it allows empathy for the parents' anxiety and sense of helplessness. Doing so can also help clarify the aspects of allergy management that are most difficult for a given family, thus guiding further intervention. 

Moreover, guidance for parents of allergic children should not be limited to a single discussion. The parents' role with respect to the child's allergy will change over time, as the child develops, so ongoing professional support and communication are needed. For example, parents must learn developmentally appropriate degrees of child independence at various ages, how best to influence child behavior at different ages (see above), and how best to advocate for one's child as he or she progresses through the school system. Policies regarding the allergic child and the use of epinephrine injectors may vary from school to school, so ongoing parental advocacy is needed. Siblings may respond adversely to the extra attention often required by the anaphylactic child [8], so parents may also need guidance on how to manage sibling interactions. Support groups related to child allergies may be helpful for some parents [16], and ongoing communication with families improves access to these and other resources. 

Furthermore, some children with anaphylactic conditions develop mental health problems that are not entirely allergy related. For example, children who exhibit anxious behaviors that predate a diagnosis of anaphylaxis may have anxiety disorders in addition to anaphylaxis-related anxiety [8]. Children with anaphylactic conditions can also have mental health problems that interfere with allergy management. For example, children with attention or learning problems may have difficulty remembering appropriate precautions or may be prone to misplacing epinephrine injectors or other allergy-related medications. Therefore, specialist referral for concurrent mental health problems can be helpful if these are present. 

## 4. Conclusions

Children and adolescents with anaphylactic conditions can learn to function well at home, at school, and socially when their anxiety is not excessive, developing into well-adjusted young adults. For this to occur, however, the physical, cognitive, and behavioral aspects of anxiety that may be associated with anaphylactic risk must be addressed, and parents must be involved in the child's care in constructive ways. Ongoing professional support and communication with these youth and their families is needed to ensure optimal psychological as well as medical outcomes. 

## Figures and Tables

**Table 1:** Key findings and recommendations of included studies.

Study	Method	Key findings	Recommendations
Akeson et al., 2007 [15]	Qualitative study of anaphylactic adolescents and their parents.	Adolescents perceived anaphylaxis as “no big deal” and could not remember a reaction; parents reported anxiety about “handing over” management of anaphylaxis to adolescents.	Tailored information for transition from parental to self-management needed; regular reviews and reinforcement about avoidance and emergency management needed; offer peer support via workshops.

Avery et al., 2003 [9]	Peanut allergic and diabetic children compared on a quality of life questionnaire.	Peanut allergic children reported lower quality of life and higher anxiety; epinephrine injectors and eating in familiar places seemed to reduce anxiety.	Anxiety may promote better adherence to allergen avoidance; epinephrine injectors may ease excessive anxiety.

Cummings et al., 2010 [10]	Nut allergic children and mothers completed questionnaires on anxiety and quality of life.	Children had lower quality of life relative to norms; mothers and children were less anxious when prescribed epinephrine injectors, regardless of their adherence to precautions.	Prescribe epinephrine injectors to reduce anxiety; provide additional education/advice to improve adherence and reduce risk taking.

DunnGalvin et al., 2009 [27]	Comparison of parents of food allergic children who enrolled child in immunotherapy study with those who did not.	Parents who enrolled their children reported higher anxiety, but similar quality of life.	Study samples may be biased towards anxious parents; avoid taking advantage of anxious parents' vulnerability when recruiting for studies.

DunnGalvin et al., 2008 [28]	Evaluation of quality of life questionnaire for parents of food allergic children.	The Food Allergy QoL-Parent Form shows excellent reliability and validity.	Consider using this questionnaire to assess health-related quality of life in parents of food allergic children.

Eigenmann et al., 2006 [25]	Survey of food allergic patients after a negative food challenge.	25% of patients continued to avoid the food, fearing persistence of allergy.	Reassess food consumption in patients with negative food challenge; repeat challenge if avoidance continues.

Friedman et al., 1994 [4]	Case series of 10 patients with recurrent unexplained flushing.	Several were originally diagnosed as anaphylactic, but eventually found to have somatization disorders.	Recognition of this presentation is needed to avoid unwarranted examinations and procedures.

Hawkes et al., 2010 [29]	Retrospective review of cases admitted to hospital for MMR immunization in Ireland.	Children often admitted due to history of egg allergy, even though risk of anaphylactic reaction is very low in this population.	Advise routine community vaccination for children with egg allergy; educate physicians about their low anaphylaxis risk.

Herbert and Dahlquist, 2008 [11]	Comparison of food allergic and nonallergic adolescents/young adults on self-report measures.	Perceived autonomy, anxiety, depression, and parental behavior did not differ between groups; those with anaphylaxis reported more worry and parental overprotection than those with less severe allergies.	Recognize that anaphylactic individuals and their parents are at particular risk for psychological distress; further study is needed.

Hu et al., 2008 [16]	Survey and qualitative interviews with parents of food allergic children.	Parents found consumer organizations good sources of practical information and support, but some nonspecific advice and contact with other anxious parents were unhelpful.	Clinicians should guide parents as to what aspects of consumer organizations are most helpful.

Khetsuriani et al., 2010 [5]	Review of adverse events in a measles-rubella vaccination campaign in Georgia.	79 severe adverse events; 37 of these had symptoms of syncope or anxiety attack, and all but one of these was initially diagnosed anaphylactic.	Risk communication strategies for care providers and the public are needed during public vaccination campaigns.

King et al., 2009 [14]	Quality of life reports from children with peanut allergy, parents, and siblings.	Mothers reported poorer quality of life and higher anxiety than fathers; separation anxiety greater in children with peanut allergy than their siblings.	Be aware that child's allergy management may fall to mothers, increasing their personal and family stress; foster allergy self-care for children to reduce anxiety.

Lebovidge et al., 2006 [12]	Development and evaluation of a questionnaire regarding parental response to children's food allergies.	Factor analysis revealed anxiety/distress, psychosocial impact of allergy, parental coping/competence, and family support factors. Greatest anxiety if child had many allergies or had anaphylaxis.	This measure may be a useful screening tool to identify parents of allergic children who are most vulnerable to anxiety and high psychosocial impact of child's allergy.

Lyons and Forde, 2004 [17]	Comparison of adolescents/young adults with/without food allergy on self-report questionnaire.	Allergy had less impact on allergic individuals' lives than others thought; allergic youth with high health competence reported greatest anxiety; few subjects knew the meaning of the term “anaphylaxis.”	Health education is needed in this population; increased vigilance among health competent individuals may increase anxiety or anxious individuals may self-diagnose food allergy; more research is needed.

Mandell et al., 2005 [2]	Qualitative interviews of parents of anaphylactic children.	Repeated cycles of adaptation to episodic anxiety-provoking (i.e., anaphylaxis-related) events challenge families to regain a sense of control.	Recognize patterns of family adaptation to anaphylaxis; help families maintain an optimal balance between protective and debilitating anxiety.

Oude et al., 2002 [23]	Randomized controlled trial of patients receiving either immunotherapy or epinephrine injector for yellow jacket allergy.	Quality of life reported as improved in immunotherapy group but not in epinephrine injector group.	Provide venom immunotherapy to improve quality of life and decrease anxiety in this population.

Powers, 2004 [6]	Single case report of reaction to jellyfish sting reported as anaphylaxis.	Individual had asthmatic attack due to anxiety induced by the jellyfish sting.	Emergency workers should treat presenting symptoms rather than assuming that anaphylaxis has occurred.

Primeau et al., 2000 [18]	Comparison of quality of life and family relations in parents of children with peanut allergy versus rheumatological disease.	Parents of peanut allergic children reported that children had more disruption in daily life and the condition had more impact on the family.	Accurate diagnosis of peanut allergy, support for families, and offering more peanut-free products would help these children and families.

Roberts-Thompson et al., 1985 [13]	Retrospective review of 98 cases of bee sting anaphylaxis.	Most reactions occurred in children; considerable anxiety present in some subjects.	Provide venom immunotherapy to alleviate anxiety.

Sampson et al., 2006 [19]	Internet questionnaire for 174 food allergic adolescents and young adults.	High-risk behavior associated with less “concern,” and with social situations involving peers.	Education of food allergic teens and also of their peers is needed to reduce risk of anaphylaxis.

Sicherer et al., 2001 [20]	Comparison of 253 parents of food allergic children versus established norms on psychosocial function questionnaire.	Low health perception of child, high emotional impact on parent, high limitation of family activities reported, especially if child had multiple food allergies.	Be aware of these psychological effects on child and family; provide family support and education; raise public awareness of the issue; advocate for food labeling.

Somers, 2011 [21]	Case report of 11-year old with peanut allergy.	Subject had very restricted diet due to fear of anaphylaxis, affecting weight gain; tense family interactions around meals.	Offer nutritional guidance; use 24-hour food recall; offer behavioral guidelines for parents; get child involved in food preparation to increase confidence.

Vargas et al., 2011 [22]	Qualitative study of parents of food allergic children.	Parents wanted (1) concise information on symptoms, cross-contamination of foods, label reading, epinephrine injectors, and advocacy; (2) education of professionals and community.	Parents of newly diagnosed children could benefit from a food allergy management curriculum; clear, concise materials would likely reduce anxiety.

Zijlstra et al., 2010 [24]	Parental anxiety measured before and after allergic children underwent food challenges.	Parental state anxiety decreased with food challenge regardless of result; parental trait anxiety was unchanged.	Food challenges may help alleviate parental anxiety about their children's allergies.
